# Evaluation of Four eGFR Calculating Formulae in Predicting Postoperative Acute Kidney Injury in Adult Patients Undergoing Open-Heart Surgery with Cardiopulmonary Bypass

**DOI:** 10.1155/2022/6929758

**Published:** 2022-07-13

**Authors:** Xiaoyun Wu, Feng Qiu, Xianglan Jin, Qiang Liu, Jian Zhou, Xia Duan

**Affiliations:** ^1^Department of CardiacSurgery, Shanghai Tenth People's Hospital, School of Medicine, Tongji University, Shanghai 200072, China; ^2^Department of Nursing, Shanghai First Maternity and Infant Hospital, School of Medicine, Tongji University, Shanghai, China

## Abstract

**Objective:**

There are four widely-used formulae to calculate the perioperative glomerular filtration rate (GFR) of patients undergoing cardiac surgery. We assessed the predictive values of these formulae in the occurrence of postoperative acute kidney injury (AKI).

**Methods:**

Patients who underwent open-heart valvular surgery with cardiopulmonary bypass from January 2015 to October 2017 were enrolled in this retrospective study. Demographic data and perioperative serum creatinine levels were collected. The estimated GFR (eGFR) was calculated using four formulae: Cockcroft Gault (CG), body surface area (BSA) corrected CG, simplified modification of diet in renal disease (MDRD), and chronic kidney disease-epidemiology collaboration (CKD-EPI) formula. The incidence of post-operative AKI was calculated and the predictive capability of these formulae was evaluated.

**Results:**

A total of 290 patients were included. 136 patients (46.90%) developed AKI after surgery. The eGFR in the AKI group was significantly lower than those in the non-AKI group at all investigated time points. In addition, the eGFR in the non-AKI group increased temporarily on the day of operation, then decreased on the following days, and returned to preoperative level about one week after surgery. However, in the AKI group, the eGFR decreased from the day of operation, which still did not recover to the preoperative level by the end of the first week after surgery. The eGFR calculated by the BSA-standardized CG formula had the highest AUC ROC curves of 0.699 and 0.774 before operation and on the day of operation, respectively. While eGFR calculated by CKD-EPI formula had the highest AUC ROC of 0.874 and 0.887 at the first and second postoperative day.

**Conclusions:**

The eGFR formula is a powerful tool for perioperative renal function assessment. The BSA-corrected CG and CKD-EPI formula have better performance in predicting postoperative AKI after cardiopulmonary bypass than serum creatinine level and other formulae.

## 1. Introduction

Acute kidney injury (AKI) is a common and serious complication after open-heart surgery with cardiopulmonary bypass (CPB) [1–3]. The known risk factors include pre-existing chronic kidney disease (CKD), age, uncontrolled hypertension, diabetes, intraoperative hypothermia, long duration of CPB, etc. It is reported that among those critically ill patients, the mortality could be as high as 50.0% [4]. Especially for patients undergoing open-heart surgery with CPB, Severe postoperative AKI often means prolonged mechanical ventilation, duration of intensive care unit (ICU), or even death. Therefore, it is widely recognized that early diagnosis is crucial to prevent postoperative AKI and improve the prognosis [5]. Serum creatinine has been applied as a classic biomarker of renal function for several decades, while due to various limitations, serum creatinine is unable to timely reflect the real status of renal function, which leads to its limited value in guiding clinical treatment. Using a specific formula to calculate the estimated glomerular filtration rate (eGFR) has been proved to be more sensitive and precise in renal function evaluation. According to the previous studies, there is no published research on the application of eGFR formulae for the early diagnosis of AKI after cardiac surgery with CPB. Therefore, we conducted this retrospective study to investigate the perioperative eGFR using four widely-used eGFR formulae, including Cockcroft Gault (CG) formula [6], body surface area (BSA) corrected CG formula, internationally common simplified modification of diet in renal disease (MDRD) formula [7] and chronic kidney disease-epidemiology collaboration (CKD-EPI) [8], and evaluate them in terms of predicting perioperative AKI at different time points.

## 2. Materials and Methods

### 2.1. Population

Patients who underwent open-heart valvular surgery with CPB in the Department of Cardiothoracic Surgery of Shanghai 10th People's Hospital Affiliated to Shanghai Tongji University from January 2015 to October 2017 were enrolled in this study.

Inclusion criteria: (1) patients aged between 18 years old and 85 years old; (2) open-heart valvular surgery with CPB.

Exclusion criteria: (1) patients aged below 18 years old or over 85 years old; (2) preoperative critical state (cardiogenic shock, malignant arrhythmia, heart dysfunction (NYHA class IV), mechanical ventilation, etc.); (3) preoperative fever, body temperature >38°C; (4) preoperative urinary system infection; (5) postoperative critical state (massive bleeding requires reoperation, malignant arrhythmia, cardiac arrest, acute cardiac tamponade); (6) emergency surgery.

This study was in accordance with the standards of medical ethics, approved by the ethics committee of the hospital (approval number: SHSYIEC-KY-4.0/16-31/01), and registered in the Chinese Clinical Trial Registry (registration number: CHICTR2000030869). All tests were conducted with the informed consent of patients or their families.

### 2.2. Data Collection

General information of patients (gender, age, height, and weight) was recorded, and BSA as well as body mass index (BMI) were calculated.

The serum creatinine level at five different time points, including before surgery, return to the ICU immediately after surgery, 1st, 2nd, and 7th days after surgery were collected. According to 2012 kidney disease improving global outcomes (KDIGO)-AKI guidelines [9], the patients were diagnosed with AKI if the serum creatinine level increased by 26.5 umol/L within 48 h postoperatively or increased over 1.5 times of preoperative baseline within 7 days postoperatively; or the postoperative urine volume was less than 0.5 ml/kg·h, lasting for 6 hours or longer (Table 1).

The eGFR of all enrolled patients at all observed time points were calculated using four widely-used creatinine clearance formulae including CG formula, BSA-corrected CG formula, internationally common simplified MDRD formula, and CDK-EPI formula.

### 2.3. Statistical Analysis

SPSS 19.0 software was applied for statistical analysis. The measurement data of normal distribution were expressed as mean ± standard deviation (SD), and the *t*-test was used for the comparisons between groups. Non-normal distribution measurement data were expressed by *M* (*Q*1, *Q*3), and the Wilcoxon test was used for comparison between groups. Counting data were obtained using the chi-square test or Fisher's exact probability. Receiver operating characteristic (ROC) curve and area under curve (AUC) were used to evaluate the diagnostic efficiency of various eGFR formulae for AKI. *P* < 0.05 was considered statistically significant.

## 3. Results

### 3.1. Basic Data

A total of 290 patients undergoing valvular surgery with cardiopulmonary bypass were enrolled in this study, including 115 male patients (39.66%). All patients were successfully returned to the ICU and 12 of them died. According to the 2012 KDIGO-AKI guidelines, 136 patients developed AKI after surgery, with an incidence of 46.90% (Figure 1). Baseline characteristics of patients are presented in Table 2. Those who develop AKI, stay longer in the ICU and require prolonged mechanical ventilation, and are also more likely to have hypoxemia, hypocardiac output syndrome (*P* < 0.001). The postoperative mortality of the AKI group was significantly increased.

### 3.2. Perioperative Serum Creatinine Expression

At all the observed time points, the serum creatinine levels of the patients in the AKI group were consistently higher than those in the non-AKI group, and the differences were statistically significant (Table 3).

The serum creatinine level of non-AKI patients decreased on the day of the operation, but increased slightly on the first day after the operation, and recovered on the 7th day after the operation. However, in the AKI group, the serum creatinine level began to increase on the day of the operation and achieved its highest level on the second day after the operation. Nevertheless, the serum creatinine level of patients in the AKI group did not recover to the preoperative level by the 7th day after the operation Table 3.

### 3.3. Changes in Perioperative eGFR Calculated by Four Different Formulae

Compared with the non-AKI group, the eGFR of the patients in the AKI group was significantly lower (*P* < 0.001) at all observed time points, regardless of different formulae (Table 4).

There are differences in the values of eGFR when different formulae are used, but the differences among these formulae are consistent in terms of groups and observed time points. The eGFR calculated by four different eGFR formulae from low to high are corrected CG formula, CG formula, MDRD, and CKD-EPI.

In non-AKI group, compared with the pre-operative level, the eGFR showed a slight increase on the day of operation but decreased to the lowest level on the first day after operation, and then gradually came back to the preoperative level on the 7th day after operation. On the other hand, the eGFR in the AKI group started to decrease on the day of operation and reached the lowest point on the second day after the operation, which did not recover by the 7th day after the operation Table 4.

### 3.4. ROC Analysis of eGFR Diagnosis of AKI

The ROC analysis of eGFR diagnosis of AKI has been shown in Table 5. The eGFR calculated by the corrected CG formula had the highest AUROC of 0.699 and 0.774 before surgery and on the day of operation, respectively, which means the best performance in predicting the development of postoperative AKI, when compared with the serum creatinine level and three other formulae.

However, on the first and second postoperative day, the eGFR calculated by the CKD-EPI formula has the best performance in predicting the development of postoperative AKI, with its AUROC at 1 and 2 days postoperatively being 0.874 and 0.887, respectively.

## 4. Discussion

AKI is a common noncardiac complication after cardiopulmonary bypass with an incidence ranging from 30% to 50% [1–9], which is an independent risk factor for postoperative death, as well. The high incidence of CPB related AKI is due to not only the ischemia/reperfusion injury during cardiopulmonary bypass, but also the presence of perioperative cardiorenal syndrome [10]. In addition, preoperative complications such as hypertension and diabetes are more common in cardiovascular patients. As a result, patients undergoing cardiac surgery with CPB are more likely to combine with early stage of hypertensive or diabetic nephropathy. Mostly they are still subclinical and cannot be identified through serum creatinine levels. Consequently, early identification of potential abnormalities of renal function in cardiac patients plays an important role in early targeted therapy and reducing the occurrence of postoperative AKI [11].

Although the serum creatinine level is still used clinically to evaluate the renal function of patients at present, its predicting value of postoperative AKI is limited due to the influence caused by various clinical factors such as hemodilution and age. GFR has been proved the best comprehensive index for evaluating renal function in both healthy and sick people [12–14]. Accurate assessment of GFR is of great significance in correctly screening high-risk patients, determining the stage of chronic kidney disease, evaluating the progression of disease and the efficacy of treatments, instruct clinical medication, as well. It is also a risk factor of postoperative AKI and death [15, 16]. However, due to severe preoperative conditions and the complications mentioned above of cardiac surgery patients, preoperative GFR test, renal imaging, and SPECT renal dynamic imaging cannot be performed routinely [17]. The formula for estimating the glomerular filtration rate was developed instead.

The aim of this retrospective study was to find out the best eGFR-calculating formula for evaluating renal function in patients undergoing cardiac surgery with cardiopulmonary bypass.

From the analysis of 290 cardiac patients, we found a consistent difference in the values of eGFR when different formulae were used regardless of groups or time points. The eGFR calculated using the CKD-EPI formula was the highest, followed by the MDRD formula and CG formula, while the eGFR calculated using the corrected CG formula was the lowest.

According to 2012 KDIGO-AKI guidelines, 136 out of 290 patients developed AKI after surgery, based on which all the enrolled patients were divided into two groups: the AKI group and the non-AKI group. The results have shown that the eGFR of patients in the AKI group was significantly lower both preoperatively and postoperatively than in the non-AKI group. The same phenomenon was observed in serum creatinine levels. In addition, the preoperative serum creatinine levels of AKI patients were normal, while the eGFR calculated by the CG formula was slightly abnormal, indicating that compared with serum creatinine level, the eGFR estimated by the formula is more sensitive in identifying preoperative chronic renal insufficiency. A temporary hyper renal function was observed in the non-AKI group on the day of operation, appearing as a slight decrease in the serum creatinine levels and increase in the eGFR, which can be attributed to the hemodilution and hemo-ultrafiltration during cardiopulmonary bypass.

The renal function of patients with postoperative AKI did not return to preoperative status by the first week after surgery, while the impact of cardiac surgery with CPB on the renal function of patients in the non-AKI group almost diminished on the 7th postoperative day. This difference may be one of the reasons that patients with AKI have prolonged hospitalization and higher hospital expenses.

The Cockcroft-Gault formula was developed in 1973 from 249 men with a creatinine clearance from 30 to 130 mL/min. Originally used to estimate creatinine clearance, it has been widely used to estimate GFR [18]. Since the deviation gradually increased with the increase of age [19], the researchers then suggested correcting it using body surface area and the consistency with the GFR measured by TC-DPTA improved after correction. The CKD-EPI formula, published in 2009, is derived from the CR results after the SCR test standard. It provides a more accurate estimate of GFR, which is applicable to a wider population and has less variation in test results, thus is recommended by the KIDGO organization to estimate GFR in adult patients with CKD [8, 19].

In our study, the methods of ROC curve and AUC were used to evaluate the diagnostic efficiency of various eGFR formulae for AKI. The results have shown that, at the first two observed time points (before surgery and the day of surgery), the eGFR calculated by the corrected CG formula had the best performance in predicting the occurrence of postoperative AKI, with the AUROC of 0.699 and 0.774, respectively, compared with serum creatinine level and other tested formulae. However, when we talk about the first and second postoperative day, the eGFR calculated by the CKD-EPI formula did best in predicting the occurrence of postoperative AKI, with the AUROC of 0.874 and 0.887, respectively. Kamaruzaman et al. [20] applied the glomerular filtration rate equation to estimate GFR in renal transplantation patients, and also found that CG and CKD-EPI had the best correlation with 51Cr-EDTA (the gold standard test for glomerular filtration rate), with a Pearson correlation coefficient of 0.733 (PGF accuracy was 80%), which is in consistent with our findings.

There are still some shortcomings in this study. Due to the limitations of patients' conditions, effective monitoring of GFR with gold standard could not be carried out, so the results need to be further studied and discussed. In addition, the application of different EGFR formulae may be affected by various factors such as ethnic differences, sample size, age distribution, sex ratio, body size and disease, so the GFR estimation formulae still need to be optimized when applied in different populations. Moreover, the continuous development of new biological markers for AKI provides broad perspective in the establishment of more effective GFR estimating formulae.

## 5. Conclusions

In conclusion, the eGFR has high sensitivity and is effective in identifying subclinical renal inefficiency and assessing renal function in cardiac surgery. All commonly used eGFR formulations predict postoperative AKI, but the BSA-corrected CG and CKD-EPI formulae are better predictors of postoperative AKI with CPB.

## Figures and Tables

**Figure 1:** Flow chart to show recruitment of patients to study. CPB, cardiopulmonary bypass; KDIGO, kidney disease improving global outcomes; AKI, acute kidney injury; eGFR, estimated glomerular filtration rate.

**Table 1:** Estimated glomerular filtration rate (eGFR) calculation formulae.

Name	Formula
CG	[140 − *A* (year old)] × *W* (kg)/[72 × 0.0113 × Scr (umol/L)] × 0.85 (*F*)
BSA corrected CG	186 × [Scr (umol/L) × 0.0113]^−1.154^ × *A* (year old)^−0.203^ × 0.742 (*F*)
CKD-EPI	141 × Min (Cr/k,1)^a^ − 1.209 × 0.993^*A*^ (*F* × 1.108), *k* = 0.9 (*M*)/0.7 (*F*), *A* = −0.411 (*M*)/−0.329 (*F*)
Simplified MDRD	186 × [Scr (umol/L) × 0.0113]^−1.154^ × *A* (year old)^−0.203^ × 0.742 (*F*)

CG, cockcroft gault; BSA, body surface area; CKD-EPI, chronic kidney disease-epidemiology collaboration; MDRD, modification of diet in renal disease; *A*, age; *W*, weight; *H*, height; *F*, female; *M*, male. BSA (m^2^) = 0.007184 × W (kg) 0.425 × H (cm) 0.725.

**Table 2:** Baseline characteristics of the population.

	Total	Non-AKI	AKI	*P* value
*N*, (%)	290	154 (53.1%)	136 (46.9%)	
Age (year)	62.0 (56.0,69.0)	58.5 (53.0,64.0)	66.0 (61.0–71.5)	<0.001
BSA (m^2^)	1.77 ± 0.19	1.75 ± 0.20	1.79 ± 0.18	0.13
BMI (kg/m^2^)	24.3 (21.9, 26.5)	24.2 (21.4, 26.2)	24.8 (22.0, 26.7)	0.39
Male, *n* (%)	115 (39.66%)	69 (44.81%)	46 (33.82%)	0.06
ICU stay (h)	117.25 ± 222.29	73.23 ± 64.30	168.73 ± 68.731	<0.001
Mechanical ventilation time (h)	45.37 ± 85.99	24.02 ± 41.98	70.34 ± 13.48	<0.001
Complications, *n* (%)				
Lung infection	29 (10%)	5 (3.25%)	24 (17.65%)	<0.001
Hypoxemia	21 (7.24%)	2 (1.3%)	19 (13.97%)	<0.001
Low cardiac output syndrome	56 (19.31%)	11 (7.14%)	45 (33.09%)	<0.001
Bleeding	10 (3.45%)	5 (3.25%)	5 (3.68%)	1.00
Cerebral stroke	3 (1.03%)	2 (1.3%)	1 (0.74%)	1.00
Sepsis shock	6 (2.07%)	2 (1.3%)	4 (2.94%)	0.57
Die	14 (4.83%)	1 (0.65%)	13 (9.56%)	<0.001

Data are expressed as mean ± SD or *n* (%). AKI, acute kidney injury; BSA, body surface area; BMI, body mass index.

**Table 3:** The expression of serum creatinine during the perioperative period.

	Basic	Surgery day	1 day after surgery	2 days after surgery	7 days after surgery
Non-AKI	73.37 (18.68)	70.85 (18.17)	79.03 (21.98)	78.25 (25.71)	69.66 (27.66)
AKI	83.65 (26.47)	89.31 (28.11)	127.04 (48.17)	143.03 (66.02)	135.43 (108.82)
*t*	−4.06	−7.00	−11.39	−10.99	−7.22
*P* value	<0.001	<0.001	<0.001	<0.001	<0.001

**Table 4:** Perioperative eGFR in two groups calculated by four formulae.

	Basic	Surgery day	1 day after surgery	2 days after surgery	7 days after surgery
CG					
Non-AKI	90.46(31.99)	93.51(33.40)	84.54(32.02)	87.00(33.91)	99.29(39.72)
AKI	76.22(26.64)	71.16(23.96)	52.74(23.13)	49.89(24.76)	61.80(31.56)
*t* value	4.13	6.58	9.69	10.43	8.93
*P* value	<0.001	<0.001	<0.001	<0.001	<0.001
Correct CG					
Non-AKI	74.27 (21.53)	76.79 (22.99)	69.22 (21.53)	71.24 (24.56)	80.89 (27.66)
AKI	61.26 (19.60)	57.55 (17.85)	42.55 (18.06)	40.15 (18.91)	49.77 (24.81)
*t* value	5.46	8.02	11.48	11.79	10.16
*P* value	<0.001	<0.001	<0.001	<0.001	<0.001
Simplify MDRD					
Non-AKI	96.27 (23.55)	100.13 (26.89)	88.79 (24.13)	91.65 (27.64)	106.54 (32.62)
AKI	84.59 (25.70)	78.40 (23.57)	55.52 (22.66)	51.13 (23.70)	67.51 (35.29)
*t* value	4.15	7.47	12.25	13.17	9.89
*P* value	<0.001	<0.001	<0.001	<0.001	<0.001
CKD-EPI					
Non-AKI	98.84 (25.70)	103.51 (29.01)	91.44 (26.98)	94.64 (30.90)	111.29 (36.28)
AKI	84.62 (28.21)	78.31 (25.45)	54.68 (24.28)	50.74 (25.39)	67.29 (37.12)
*t* value	4.66	8.02	12.32	12.97	10.33
*P* value	<0.001	<0.001	<0.001	<0.001	<0.001

**Table 5:** ROC analysis of eGFR diagnosis of AKI.

Index	Cutoff	AUC (95% CI)	Sensitivity (95% CI)	Specificity (95% CI)
Before surgery				
Creatinine	91.00	0.623 (0.558–0.688)	0.346 (0.266, 0.426)	0.857 (0.802, 0.912)
CG	85.23	0.658 (0.595–0.721)	0.728 (0.653, 0.803)	0.552 (0.473, 0.631)
Correct CG	66.42	0.699 (0.639–0.760)	0.691 (0.614, 0.769)	0.643 (0.567, 0.719)
Simplify MDRD	88.66	0.648 (0.584–0.712)	0.588 (0.506, 0.671)	0.682 (0.608, 0.755)
CKD-EPI	92.39	0.673 (0.611–0.735)	0.662 (0.582, 0.741)	0.643 (0.567, 0.719)
Surgery day				
Creatinine	67.70	0.721 (0.663–0.780)	0.831 (0.768, 0.894)	0.533 (0.454, 0.611)
CG	78.47	0.737 (0.679–0.794)	0.684 (0.606, 0.762)	0.682 (0.608, 0.755)
Correct CG	66.59	0.774 (0.720–0.828)	0.779 (0.710, 0.849)	0.675 (0.601, 0.749)
Simplify MDRD	90.71	0.743 (0.687–0.799)	0.750 (0.677, 0.823)	0.623 (0.547, 0.700)
CKD-EPI	97.73	0.761 (0.706–0.815)	0.831 (0.768, 0.894)	0.571 (0.493, 0.650)
1 day				
Creatinine	90.90	0.854 (0.809–0.899)	0.802 (0.734, 0.869)	0.773 (0.707, 0.839)
CG	59.34	0.840 (0.793–0.887)	0.728 (0.653, 0.803)	0.838 (0.779, 0.896)
Correct CG	54.37	0.871 (0.829–0.914)	0.838 (0.776, 0.900)	0.779 (0.714, 0.845)
Simplify MDRD	67.30	0.869 (0.827–0.912)	0.7647 (0.693, 0.836)	0.857 (0.802, 0.912)
CKD-EPI	70.83	0.874 (0.832–0.916)	0.824 (0.759, 0.888)	0.805 (0.743, 0.867)
2 days				
Creatinine	99.10	0.872 (0.830–0.914)	0.735 (0.661, 0.809)	0.903 (0.856, 0.949)
CG	61.74	0.846 (0.799–0.893)	0.802 (0.734, 0.869)	0.786 (0.721, 0.851)
Correct CG	50.40	0.875 (0.832–0.918)	0.802 (0.734, 0.869)	0.812 (0.750, 0.873)
Simplify MDRD	68.73	0.891 (0.851–0.931)	0.838 (0.776, 0.900)	0.805 (0.743, 0.868)
CKD-EPI	65.99	0.887 (0.847–0.928)	0.809 (0.743, 0.875)	0.831 (0.772, 0.890)

## Data Availability

The data used to support the findings of this study are available from the corresponding author upon request.
